# Fenofibrate plus Metformin Produces Cardioprotection in a Type 2 Diabetes and Acute Myocardial Infarction Model

**DOI:** 10.1155/2016/8237264

**Published:** 2016-03-16

**Authors:** Víctor Hugo Oidor-Chan, Enrique Hong, Francisca Pérez-Severiano, Sergio Montes, Juan Carlos Torres-Narváez, Leonardo del Valle-Mondragón, Gustavo Pastelín-Hernández, Alicia Sánchez-Mendoza

**Affiliations:** ^1^Department of Pharmacobiology, Research and Advanced Studies Center, National Polytechnic Institute (IPN), Calzada de los Tenorios No. 235, Colonia Granjas Coapa, Tlalpan, 14330 Mexico City, Mexico; ^2^Department of Pharmacology, National Institute of Cardiology Ignacio Chávez, Juan Badiano No. 1, Colonia Sección XVI, Tlalpan, 14080 Mexico City, Mexico; ^3^Department of Neurochemistry, National Institute of Neurology and Neurosurgery Manuel Velasco Suárez, Insurgentes Sur No. 3877, Colonia La Fama, Tlalpan, 14269 Mexico City, Mexico

## Abstract

We investigated whether fenofibrate, metformin, and their combination generate cardioprotection in a rat model of type 2 diabetes (T2D) and acute myocardial infarction (AMI). Streptozotocin-induced diabetic- (DB-) rats received 14 days of either vehicle, fenofibrate, metformin, or their combination and immediately after underwent myocardial ischemia/reperfusion (I/R). Fenofibrate plus metformin generated cardioprotection in a DBI/R model, reported as decreased coronary vascular resistance, compared to DBI/R-Vehicle, smaller infarct size, and increased cardiac work. The subchronic treatment with fenofibrate plus metformin increased, compared with DBI/R-Vehicle, total antioxidant capacity, manganese-dependent superoxide dismutase activity (MnSOD), guanosine triphosphate cyclohydrolase I (GTPCH-I) expression, tetrahydrobiopterin : dihydrobiopterin (BH_4_ : BH_2_) ratio, endothelial nitric oxide synthase (eNOS) activity, nitric oxide (NO) bioavailability, and decreased inducible NOS (iNOS) activity. These findings suggest that PPAR*α* activation by fenofibrate + metformin, at low doses, generates cardioprotection in a rat model of T2D and AMI and may represent a novel treatment strategy to limit I/R injury in patients with T2D.

## 1. Introduction

Type 2 diabetes (T2D) is a chronic metabolic disorder that results from defects in both insulin secretion and insulin action. Elevated rates of basal hepatic glucose production in the presence of hyperinsulinemia are the primary cause of fasting hyperglycemia; after a meal, impaired suppression of hepatic glucose production by insulin and decreased insulin-mediated glucose uptake by muscle contribute almost equally to postprandial hyperglycemia [1]. Diabetic patients develop vascular complications at a much faster rate in comparison to nondiabetic individuals, and cardiovascular risk is increased up to tenfold [2]. It is estimated that more than 50% of diabetic patients die from a cardiovascular event, most likely coronary artery disease [3]. The development of cardiovascular disease in T2D is multifactorial; some mechanisms include glucose itself as well as glucose dependent mechanisms, such as the formation of advanced glycation end-products (AGEs) [4], the activation of vasoactive hormonal systems, for example, the renin-angiotensin system (RAS) [5], and increased oxidative stress [4].

Under physiological conditions, in the vasculature, nitric oxide (NO) is produced mainly by endothelial nitric oxide synthase (eNOS), where it fulfills vasodilatory, antithrombotic, and antiatherosclerotic functions [6]. However, in pathological conditions, such as T2D [7] and acute myocardial infarction (AMI) [8], NO bioavailability in the vasculature decreases and eNOS becomes uncoupled producing superoxide anion instead of NO [6]. A major cause for eNOS uncoupling is likely to be a deficiency of the NOS cofactor tetrahydrobiopterin (BH_4_) [9]. Under pathological conditions, associated with increased oxidative stress, superoxide anion and peroxynitrite can oxidize BH_4_, leading to BH_4_ deficiency [10].

Peroxisome proliferator-activated receptors (PPARs) belong to a subfamily of the nuclear receptors involved in glucose and lipid metabolism; the group includes three isotypes encoded by different genes: PPAR*α*, PPAR*β*/*δ*, and PPAR*γ* [11]. PPAR*α* was the first to be discovered and it causes cellular peroxisome proliferation in rodent liver [12], giving this receptor family its name. PPAR*α* is highly expressed in the heart, liver, kidney, intestine, and brown adipose tissue, all of which are characterized by an elevated rate of fatty acid catabolism [11]. Recently, in our laboratory we observed that the stimulation of PPAR*α* with clofibrate restores eNOS function and decreases oxidative stress in a rat model of hypertension secondary to aortic coarctation (AoCo) [13]. Moreover, it has been observed that PPAR*α* ligands, including fibrates, reduce myocardial ischemia/reperfusion (I/R) injury in diabetic and nondiabetic animals; this cardioprotection might be mediated through anti-inflammatory mechanisms and via the activation of the phosphatidylinositol-4,5-bisphosphate 3-kinase (PI3K)/protein kinase B (Akt)/NO pathway [8, 14, 15]. Recently, Barreto-Torres et al. [16] showed that metformin, a widely used antidiabetic drug for T2D, exerts cardioprotection in rats with myocardial I/R injury via activation of PPAR*α*.

Therefore, the aim of this work was to test whether the PPAR*α* activators fenofibrate and metformin and/or their combination exerts an antioxidant effect and preserves NO production leading to cardioprotection. We also aimed to evaluate the effectiveness of the treatments producing cardioprotection in a rat model of T2D and AMI.

## 2. Material and Methods

All animal procedures were conducted in accordance with Federal Regulations concerning Animal Experimentation and Care (Ministry of Agriculture, SAGARPA, NOM-062-ZOO-1999, Mexico). Animal protocol experimentation was approved by the Ethical Committee of our institution (CICUAL, Protocol 502-12) and conducted according to the Guidelines for Care and Use of Experimental Animals.

### 2.1. Animals

Neonate male Wistar rats (3-4 days old) were divided into 2 groups. Control- (CT-) rats received 0.1 M citrate buffer, pH 4.5 (vehicle), intraperitoneally (i.p.); and diabetic- (DB-) rats received a single streptozotocin (STZ) dose in vehicle (70 mg/kg, i.p.). Body weight and blood glucose levels were measured weekly during 8 weeks. Blood from the tail was collected for capillary glucose determination in fasted and nonfasted rats using a glucometer (Accu-Chek Active, Glucotrend, Roche®). Eight weeks after STZ administration, we conducted an oral glucose tolerance test (OGTT) and determined insulin secretion (these tests were performed with 14 hours of fasting). At this stage, animals from both experimental groups were randomly subdivided to receive one of the subchronic (14 days) oral treatments: (a) vehicle (NaCl 0.9%), (b) fenofibrate (100 mg/kg), (c) metformin (100 mg/kg), (d) metformin (300 mg/kg), or (e) fenofibrate (50 mg/kg) + metformin (50 mg/kg). At the end of the treatment, rats were assigned to either sham-operation or myocardial ischemia for 30 min followed by 120 min of reperfusion.

### 2.2. Acute Myocardial Infarction in Rats

At the end of the subchronic treatment, the rats were anesthetized with a combination of ketamine hydrochloride (80 mg/kg, i.m.) and xylazine hydrochloride (10 mg/kg, i.m.). The animals were intubated and artificially ventilated (50 strokes/min, 8–10 mL/kg tidal volume). A left intercostal thoracotomy was performed to expose the heart; subsequently myocardial ischemia was induced by the occlusion of the left anterior descending coronary artery (LAD) with a 6-0 silk suture through myocardial tissue. After 30 min of ischemia, the occlusion was released and the myocardium was reperfused for 120 min. Control animals (sham-operation) were treated in a similar fashion, except for LAD tie.

### 2.3. Determination of Infarct Size

After 120 min of reperfusion, the LAD was reoccluded and 1.5 mL of 2% Evans blue dye was injected into the right atrium via the left jugular vein to outline the ischemic myocardium (area at risk). The rats were euthanized and the hearts were rapidly excised. The hearts were frozen at −20°C for 1 hour and then cross sections of 2 mm thickness were performed. The slices were incubated with 2,3,5-triphenyltetrazolium hydrochloride at 1% in phosphate buffer (0.1 M, pH 7.4) for 15 min at 37°C to distinguish the viable myocardium from the necrotic. After overnight incubation in 10% formalin, the slices were scanned from both sides and weight was obtained. The extent of myocardial necrosis and the area at risk were determined by planimetry (Image J).

### 2.4. *Ex Vivo* Cardiac Function Evaluation

After subchronic treatment and sham or I/R, the hearts of CT- and DB-rats were excised, rapidly cannulated retrogradely through the ascending aorta onto a Langendorff system, and perfused with Krebs-Henseleit buffer (37°C) saturated with 95% O_2_/5% CO_2_ at 12 mL/min constant flow rate. The Krebs-Henseleit buffer consisted of the following (in mM): 117.8 NaCl, 1.2 NaH_2_PO_4_·H_2_O, 0.027 EDTA, 6.0 KCl, 1.6 CaCl_2_·2H_2_O, 1.2 MgSO_4_·7H_2_O, 25 NaHCO_3_, and 5.55 dextrose pH 7.4. A latex balloon, connected to a pressure transducer (Statham 7320, Statham Instruments, Inc., Hato Rey, Puerto Rico), was inserted into the left ventricle through an incision in the left atrium. The balloon was then filled with Krebs-Henseleit buffer at 10 mmHg steady diastolic pressure. The function of this balloon is to measure the left ventricular pressure (LVP). Coronary perfusion pressure (PP) was measured by means of a pressure transducer (Gould P23ID, Gould Instruments, Cleveland, OH) at the level of the right and left ostium. The heart rate was maintained constant by stimulation with an epicardial ventricular pacemaker (Grass-SIU5, Grass Instruments Co.), to reach 312 beats/min (5 Hz). The heart was stabilized for 30 min and the following hemodynamic parameters were monitored using a computer acquisition data system (Grass 79D, Grass Instruments Co., Quincy, MA): coronary vascular resistance (CVR) was obtained calculating the ratio between PP (mmHg) and flow rate (mL/min) and mechanical work was obtained as the product of LVP (mmHg) × heart rate (beats/min).

### 2.5. Western Blot

Thirty micrograms of protein from myocardial ischemic areas from the different experimental groups was separated on sodium dodecyl sulfate/polyacrylamide gel, transferred to polyvinylidene difluoride membranes, and then blocked with 8% skim milk in phosphate-buffered saline pH 7.4. The membranes were incubated overnight at 4°C with specific antibodies against PPAR*α* (1 : 1000, Santa Cruz Biotechnology, Santa Cruz, CA), guanosine triphosphate cyclohydrolase I (GTPCH-I) (1 : 1000, Santa Cruz Biotechnology, Santa Cruz, CA), eNOS (1 : 5000, Santa Cruz Biotechnology, Santa Cruz, CA), or *β*-actin (1 : 20000, Millipore, Darmstadt, Ger). The membranes were incubated for 1 h at room temperature with their corresponding secondary antibody: goat anti-mouse (1 : 15000, Jackson ImmunoResearch, PA, USA), goat anti-mouse (1 : 5000, Jackson ImmunoResearch), donkey anti-goat (1 : 5000, Jackson ImmunoResearch, PA, USA), or goat anti-mouse (1 : 40000, Jackson ImmunoResearch, PA, USA). Blots were washed and visualized using a chemiluminescence kit (Immobilon Western, Millipore, MA, USA). Bands were detected employing a ChemiDoc XRS+ system (BIO-RAD, USA). The bands were quantified by densitometry employing the Image Lab 5.0 software. The results are expressed as arbitrary units (AU) of the ratio between protein and *β*-actin.

### 2.6. Measurement of Total Antioxidant Capacity

Total antioxidant capacity (TAC) in serum was determined as previously reported by Ibarra-Lara et al. [17]. Briefly, in a 96-well plate 35 *μ*L of serum was placed with 145 *μ*L of 0.1 M phosphate buffer pH 7.5 and homogenized at 500 rpm for 200 s. Immediately after, 100 *μ*L of diluted serum was transferred to the adjacent well, mixed with 50 *μ*L CuCl_2_ 0.01 M, and homogenized at 500 rpm for 200 s. Finally, 50 *μ*L bathocuproine 0.01 M was added and mixed (500 rpm/200 s). Samples were read at 490 nm excitation and 190 nm emission. TAC is expressed as *μ*mol/L of Cu^2+^ reduced to Cu^+^.

### 2.7. Superoxide Dismutase Activity

The superoxide dismutase (SOD) activity was determined by the method described by Flohé and Otting [18]. Myocardial ischemic areas from the different experimental groups were homogenized in a buffer consisting of 20 mM sodium bicarbonate, 0.02% Triton X-100, pH 10.2. Twenty *μ*L of clarified supernatant from homogenized samples was added to 2.85 mL of reaction mixture containing 10 *μ*M cytochrome C, 10 *μ*M sodium azide, 100 *μ*M xanthine, and 1 mM EDTA in 20 mM sodium bicarbonate, 0.02% Triton X-100, pH 10.2. The assay was initiated by adding xanthine oxidase. The mixture was homogenized and absorbance determined spectrophotometrically at 550 nm every 30 seconds for 3 minutes. The activity of manganese SOD (MnSOD) was measured in the same manner as total SOD activity, but the reaction was incubated with 50 *μ*L of KCN (1 mM) to inhibit Cu/ZnSOD. The difference between total SOD and MnSOD represents Cu/ZnSOD activity. Results are expressed as SOD units/mg protein. One unit of SOD is defined as the amount of enzyme that inhibits at 50% the rate of cytochrome c reduction, under specified conditions.

### 2.8. Determination of BH_4_ and BH_2_ Production

The production of BH_4_ and BH_2_ was determined as previously reported by Cervantes-Pérez et al. [13]. Briefly, myocardial ischemic areas from different experimental groups were analyzed by capillary zone electrophoresis (CZE, P/ACE MDQ Capillary Electrophoresis System, Beckman Coulter, Inc., Fullerton, CA, USA) to measure BH_4_ and BH_2_ simultaneously. Capillary electrophoretic separation was achieved using a Sep-Pak® Aminopropyl (NH2) Classic Cartridge. Sample separation was performed by applying 30 kV for 10 min and UV determination was at 230 nm. Data are expressed as pmol of BH_4_ or BH_2_ per mg of wet tissue.

### 2.9. NOS Activity Determination

Quantification of NOS activity was measured according to Ibarra-Lara et al. [17]. The basis of the technique involved the conversion of L-[^3^H]-arginine into NO and L-[^3^H]-citrulline, in the presence of the appropriate enzyme cofactors.

### 2.10. Quantification of NO in Biological Samples

The NO production in myocardial ischemic areas from different experimental groups was evaluated using the technique described by Griess and modified by Tenorio and del Valle [19].

### 2.11. Statistical Analysis

Results are expressed as mean ± standard error of the mean (SEM). Experimental data were examined employing the two-way ANOVA followed by Duncan's* post hoc* test. Statistical significance was set at *P* < 0.05. All analyses were carried out using the statistical package Sigma Plot version 12.0 (San Jose, CA, USA).

## 3. Results

### 3.1. T2D Model

Capillary glucose was determined in fasted and nonfasted rats. In fasting conditions no changes in capillary glucose were observed in CT- or DB-rats (Figure 1(a)), whereas, in nonfasting conditions, DB-rats displayed hyperglycemia compared with the CT group. Regarding body weight, DB-rats showed lower body weight compared to CT-rats (Figure 1(b)). At 8 weeks, DB-rats showed impaired glucose tolerance after glucose load (Figure 1(c)) and insulin secretion was lower compared with the CT group (Figure 1(d)).

Subchronic treatments (14 days) promoted a decrease in body weight in CT-rats (Figure 2(a)). In DB-rats none of the pharmacological treatments modified body weight (Figure 2(a)). Metformin (300 mg/kg) and the combination of fenofibrate (50 mg/kg) plus metformin (50 mg/kg) promoted the use of glucose in DB-rats, observed as a decrease in the hyperglycemia (Figure 2(b)). However, none of the pharmacological treatments (fenofibrate, metformin, or their combination) decreased glucose intolerance (Figure 2(c)).

### 3.2. Hemodynamics

We observed that I/R increased CVR (Figure 3(a)) and decreased cardiac work (Figure 3(b)) in both CT- and DB-rats; CVR was higher in DBI/R rats than in CTI/R rats. Fenofibrate and metformin (100 and 300 mg/kg) decreased CVR and increased cardiac work in both CTI/R and DBI/R rats. Interestingly, the combination exerted synergism observed as decreased CVR and increased cardiac work when compared to controls.

### 3.3. Infarct Size

No changes in the area at risk were observed among the different groups (Figures 4(a) and 4(b)), suggesting that the LAD's ligation was consistently performed at the same place. Even so, infarct size was greater in DBI/R than in CTI/R rats treated with vehicle. All treatments promoted cardioprotection in CTI/R rats observed as decreased infarct size compared with vehicle-treated CTI/R group. Cardioprotection was also exerted, by the treatments, in DBI/R compared with the DBI/R-Vehicle group. Interestingly, the combination of treatments produced cardioprotection comparable to higher doses of individual treatments (Figure 4(c)).

### 3.4. PPAR*α* Expression

Our results show that I/R decreased PPAR*α* expression in CT- and DB-rats. In DBI/R, fenofibrate and metformin (100 and 300 mg/kg) restored PPAR*α* expression to control values. In CTI/R treatments did not modify the PPAR*α* expression. Even though no statistical difference was found in DBSH-rats, a clear tendency of increased PPAR*α* expression is observed in fenofibrate- and metformin- (100 and 300 mg/kg) treated rats (Figures 5(a) and 5(b)).

### 3.5. Total Antioxidant Capacity

As shown in Figure 6, I/R and DB lowered the TAC; this event was prevented by fenofibrate and metformin in CTI/R. In terms of nonischemic DB-rats, treatments did not affect the TAC. The combination of treatments increased the TAC in I/R, DBSH, and DBI/R groups compared to control values.

### 3.6. SOD Activity

With respect to Cu/ZnSOD activity, metformin (100 and 300 mg/kg) promoted an increase only in DBI/R rats compared to the DBI/R-Vehicle group (Figure 7(a)). In DB-rats, MnSOD activity decreased in both sham- and I/R-subjected rats treated with vehicle compared to CTSH-Vehicle. Fenofibrate (100 mg/kg) increased the MnSOD activity in DBSH- and DBI/R rats compared to those treated with vehicle. While metformin (100 mg/kg) enhanced MnSOD activity only in DBI/R conditions, metformin (300 mg/kg) improved it also in CTI/R and DBI/R conditions. Interestingly, the combination of treatments increased the MnSOD activity in every experimental group (Figure 7(b)).

### 3.7. GTPCH-I Expression and BH_2_, BH_4_ Production

The expression of GTPCH-I decreased in CTI/R compared with CTSH-Vehicle. In DBSH-rats, none of the treatments significantly altered the expression of GTPCH-I. Fenofibrate and metformin (100 and 300 mg/kg) increased GTPCH-I expression in CTI/R and DBI/R groups. Interestingly, the combination of treatments (at lower doses than individually administered) increased GTPCH-I expression in both CTI/R and DBI/R groups (Figure 8(a)). Due to the high relevance of BH_4_ as a cofactor for eNOS to produce NO, we measured BH_4_ : BH_2_ ratio. As shown in Figure 8(b), I/R and DB decreased BH_4_ : BH_2_ ratio. In DBSH-rats, none of the treatments significantly modified the BH_4_ : BH_2_ ratio. However, fenofibrate and metformin (100 and 300 mg/kg), as well as the combination of fenofibrate and metformin, increased BH_4_ : BH_2_ ratio in CTI/R and DBI/R groups (Figure 8(b)).

### 3.8. eNOS Expression and NOS Activity

Our data show that eNOS expression remained comparable among groups, regardless of the treatments (Figure 9(a)). Endothelial NOS activity diminished in the left ventricular ischemic zone in response to both I/R and DB. Fenofibrate and metformin (100 and 300 mg/kg) increased eNOS activity in both CTI/R and DBI/R rats. In DBSH, none of the treatments significantly modified eNOS activity. The administration of fenofibrate + metformin improved the activity of eNOS bringing values closer to those of controls (Figure 9(c)). Since iNOS plays an important role in numerous pathophysiological conditions, for example, I/R and DB, we measured its activity. Our results show that I/R and DB increased iNOS activity, fenofibrate was able to prevent the rise in iNOS activity in DB, and metformin and the combination of treatments prevented the activation of iNOS in I/R and DB groups (Figure 9(d)).

### 3.9. NO Production

The data show that NO production decreased in the left ventricles from rats under I/R and DB conditions. Fenofibrate, metformin (100 and 300 mg/kg), and their combination prevented the NO reduction in CTI/R and DBI/R groups. However, none of the treatments significantly modified the NO production in DBSH-rats (Figure 9(b)).

## 4. Discussion

We demonstrated that fenofibrate, metformin, and the combination of treatments, at low doses, generate cardioprotection in an experimental model of T2D subjected to I/R. Pharmacological treatments prevented the rise in CVR, decreased cardiac output, and decreased infarct size; those effects were most probably achieved through the activation of PPAR*α* which promoted an antioxidant effect preserving NO bioavailability therefore improving endothelial functioning.

It has been shown that PPAR*α* expression is downregulated by chronic diabetes stressors [20] and hypoxia inducible factor-1 (HIF-1) [21]. According to that reported, we observed that, in DBSH and DBI/R subjects, the expression of PPAR*α* decreases compared with the CTSH-Vehicle group. Interestingly, in fenofibrate- and metformin-treated DBSH-rats there is a clear tendency to raise PPAR*α* expression compared with DBSH-Vehicle. The combination of treatments did not modify PPAR*α* expression in DBI/R group compared to vehicle-treated rats. This lack of stimulation for protein expression could be due to the low dose; however it was sufficient to promote cardioprotective effects.

T2D is associated with increased cardiovascular disease rates, raising the risk of myocardial infarction [2]. Patients with T2D exhibit several abnormalities in left ventricular function and impaired cardiac contractility, including reduced stroke volume, elevated end-diastolic pressure, shortened ejection time, and prolonged preejection period [22]. Interestingly, in the neonatal streptozotocin-treated rat (n-STZ) model, the extent to which cardiac performance is affected appears to be dependent on the duration of STZ treatment. Schaffer et al. [23] demonstrated that at 4 months there appears to be no mechanical dysfunction; however, at 8 and 12 months diabetic hearts showed significantly depressed cardiac function, observed as decreased aortic output, decreased ventricular pressure, and decreased cardiac work. With respect to cardiovascular hemodynamics, we did not observe changes in the CVR and cardiac work in 10-week-old DBSH-rats, probably due to animals' age and chronicity of the pathology of the DB-rats. However, after an ischemic insult, DBI/R rats exhibit increased CVR, decreased cardiac work, and increased infarct size compared to nondiabetic rats resembling T2D patients who experience a more adverse outcome after acute myocardial infarction compared with nondiabetic patients [24]. Our study demonstrates that the PPAR*α* activators fenofibrate and metformin and the combination of treatments generate cardioprotection preventing the increase of CVR and the decreased cardiac output as well as decreasing infarct size. Our research is the first study to demonstrate that the combination of fenofibrate and metformin, at low doses, generates cardioprotection probably by the activation of PPAR*α*.

Pharmacological stimulation of PPAR*α* elicits a wide array of effects. It has been reported that PPAR*α* agonists increase sensitivity to insulin-stimulated glucose uptake to a substantial degree in animal insulin resistance models and in* ex vivo* human muscle cells studies [25]. However, Rieusset et al. [26] reported that in human subjects with T2D there was no difference in insulin sensitivity after subchronic treatment with fenofibrate compared with control. Our results agree with Rieusset, since no evidence of decreased hyperglycemia or improvement in glucose tolerance in DB-rats, after a subchronic treatment with a selective PPAR*α* agonist (fenofibrate) compared with CT-rats, was observed, suggesting that the cardioprotector effect is not due to glucose lowering effect. Moreover, metformin, the first-line pharmacological treatment in the management of T2D, reported to improve glycemic control [27], at a dose of 100 mg/kg, did not improve the glucose tolerance in DB- compared with CT-rats. In our study, the subchronic treatment with fenofibrate and metformin, at low doses, lowers the hyperglycemia but does not improve the glucose tolerance in DB-rats compared with CT-rats, an effect most probably mediated by PPAR*α*.

Although the effects of fenofibrate are classically mediated via activation of PPAR*α*, several studies have demonstrated PPAR*α*-independent effects. Likewise, fenofibrate is able to exert anti-inflammatory [28, 29], antifibrotic [30], antihyperthrophic [31], and proapoptotic [32] effects in a PPAR*α*-independent way. Similarly, metformin is capable of interaction with several molecular targets including the activation of the reperfusion injury salvage kinase (RISK) pathway [33], by increasing AMPK activation [34] or via adenosine receptor stimulation [35], both of them actions that inhibit the mitochondrial permeability transition pore (mPTP) opening at reperfusion exerting cardioprotection.

We propose that fenofibrate and metformin activate PPAR*α* generating cardioprotection against I/R injury in n-STZ model, through a mechanism that involves decreased oxidative stress and increased NO bioavailability. We based our hypothesis on current and previous data reporting that clofibrate lowers oxidative stress, enhances NO bioavailability, and improves ultrastructure and ventricular hemodynamics in no-flow myocardial ischemia in rats [17]. Further, numerous studies have demonstrated cardioprotective effects of NO during I/R in T2D and nondiabetic models [8, 36, 37]. It is widely reported that NO possesses a number of physiological properties, such as vasodilation, inhibition of oxidative stress, platelet aggregation, leukocyte chemotaxis, and apoptosis, which make it a potent cardioprotective-signaling molecule [9, 10]. Under pathological conditions, such as T2D [7] and AMI [8], NO bioavailability in the vasculature decreases and eNOS becomes uncoupled producing superoxide anion instead of NO, increasing oxidative stress and leading to endothelial dysfunction [6]. In accordance with the literature, we observed that, in AMI (I/R) and T2D, parameters like NO bioavailability, MnSOD activity, and the total antioxidant capacity decreased. We also showed that fenofibrate + metformin prevented those changes in CTI/R and DBI/R. Regarding the increased bioavailability of NO, it is most probably due to increased eNOS activity, since we observed a raise in this parameter, no change in eNOS expression was observed, and previous data have shown that PPAR*α* stimulation promotes eNOS phosphorylation at Ser1177 [7].

Endothelial NOS strictly requires BH_4_ in order to be coupled and produce NO [10]. Deficient BH_4_ levels in several* in vitro* and* in vivo* models have correlated with low NO production [38]. Therefore, BH_4_ availability is a critical determinant of eNOS regulation in several pathologies (e.g., atherosclerosis) and it is a rational therapeutic target to restore NO-mediated endothelial function and reduce disease progression [39]. In our investigation, we observed that the BH_4_ : BH_2_ ratio decreased in CTI/R and DBI/R and that the treatment with agonists of PPAR*α* (fenofibrate + metformin) promoted an increase in BH_4_ : BH_2_ ratio under these conditions.

Biosynthesis of BH_4_ occurs mainly via* de novo* pathway [38]. The synthesis of BH_4_ by this pathway is initiated by the action of GTPCH-I, which is the rate-controlling enzyme. Cai et al. [40] demonstrated that the transfection of human aortic endothelial cells with GTPCH-I markedly augmented BH_4_ levels, increased total eNOS activity, increased the quantity of dimerised eNOS, and increased NO synthesis. Several studies have shown that diabetes reduces BH_4_ bioavailability by increasing 26S proteasome-dependent degradation of GTPCH-I [41]. In contrast, cardiomyocyte-specific overexpression of the GTPCH-I gene restored the efficacy of ischemic preconditioning to reduce myocardial I/R injury during hyperglycemia by increasing bioavailability of BH_4_ and NO [42]. We measured the* in vivo* expression of GTPCH-I and showed that, in I/R and DB conditions, the expression of the enzyme is decreased and the combined treatment promoted higher GTPCH-1 expression, further supporting Liu et al. [43] report showing that, in HUVECs, fenofibrate increased GTPCH-I expression in a concentration dependent manner.

At the clinical level, fenofibrate, metformin, and/or their combination have been used to treat lipid and glucose metabolic alterations [44], to study the effect on lymphocyte cytokine release in patients with early glucose metabolism abnormalities [45], and to explore the effect on coagulation and fibrinolysis in impaired glucose tolerance patients [46]. The widespread use in clinic and our data allowed us to suggest that the therapeutic effects produced by fenofibrate + metformin could exert a cardioprotector effect in T2D patients.

## 5. Conclusions

In our study we demonstrated that fenofibrate + metformin, at low doses, generates cardioprotection in a rat model of T2D and AMI most probably through PPAR*α* activation. These findings may represent a novel treatment strategy to limit I/R injury in patients with T2D.

## Figures and Tables

**Figure 1:** Characteristics of neonatal streptozotocin-induced T2D rat model. Time-course of (a) capillary glucose concentrations and (b) body weight from control- (CT-) and diabetic- (DB-) rats. (c) Capillary glucose levels and (d) serum insulin concentrations before and during an oral glucose tolerance test (OGTT) (2 g/Kg) in 8-week-old CT- and DB-rats. ^A^ *P* < 0.05 versus CT nonfasting, ^B^ *P* < 0.05 versus DB fast, and ^C^ *P* < 0.05 versus control two-way ANOVA followed by Duncan's* post hoc* test.

**Figure 2:** Effect of subchronic treatment (14 days) of different drugs on (a) body weight and (b) nonfasting capillary glucose concentrations of control- (CT-) and diabetic- (DB-) rats. (c) Capillary glucose levels in CT- and DB-rats before and during an oral glucose tolerance test (OGTT) (2 g/kg) after 14 days of subchronic treatment. (d) Area under the curve for OGTT. ^A^ *P* < 0.05 versus CT, ^B^ *P* < 0.05 versus CT-vehicle, ^C^ *P* < 0.05 versus DB-vehicle, ^E^ *P* < 0.05 versus fenofibrate (Feno, 100 mg/kg), and ^F^ *P* < 0.05 versus metformin (Metfor, 100 mg/kg) two-way ANOVA followed by Duncan's* post hoc* test. Data are presented as means ± SEM of 6 animals per group.

**Figure 3:** Evaluation of the* ex vivo* cardiac hemodynamics in control-ischemia/reperfusion (CTI/R) and diabetic-ischemia/reperfusion (DBI/R) conditions. (a) Coronary vascular resistance and (b) rate-pressure product were both measured* ex vivo* by Langendorff technique. ^A^ *P* < 0.05 versus control-sham- (CTSH-) Vehicle, ^B^ *P* < 0.05 versus diabetic-sham- (DBSH-) Vehicle, ^C^ *P* < 0.05 versus CTI/R-Vehicle, and ^D^ *P* < 0.05 versus DBI/R-Vehicle two-way ANOVA followed by Duncan's* post hoc* test. Data are presented as means ± SEM of 6 animals per group.

**Figure 4:** Subchronic treatment with fenofibrate (F), metformin (M), and their combination reduced infarct size in control-ischemia/reperfusion (CTI/R) and diabetic-ischemia/reperfusion (DBI/R) conditions. (a) Representative photographs of Evans blue/triphenyltetrazolium chloride dyed heart slices from CTI/R and DBI/R rats, the blue area represents the area with viable tissue, the red area is the area at risk (AAR), and the white regions are the necrotic areas (NA). (b) Area at risk and (c) infarct size of the different groups, expressed as a percentage of AAR in the left ventricle and percentage of NA in the AAR, respectively. ^C^ *P* < 0.05 versus CTI/R-Vehicle and ^D^ *P* < 0.05 versus DBI/R-Vehicle two-way ANOVA followed by Duncan's* post hoc* test. Data are presented as means ± SEM of 4–6 animals per group.

**Figure 5:** Subchronic treatment with fenofibrate (F), metformin (M), and their combination prevented the decreased expression of PPAR*α* in diabetic-ischemia/reperfusion (DBI/R) conditions. (a) Representative immunoblot and (b) PPAR*α* expression in ischemic left ventricle area (*n* = 4 rats/group). ^A^ *P* < 0.05 versus control-sham- (CTSH-) Vehicle and ^D^ *P* < 0.05 versus DBI/R-Vehicle two-way ANOVA followed by Duncan's* post hoc* test. Data are presented as means ± SEM.

**Figure 6:** Effect of fenofibrate, metformin, and fenofibrate + metformin on serum antioxidant capacity. Total antioxidant capacity was evaluated in serum from control- (CT-) and diabetic- (DB-) rats subjected to sham- (SH-) or ischemia/reperfusion- (I/R-) myocardial infarction and treated subchronically (14 d) with either vehicle, fenofibrate (Feno, 100 mg/kg), metformin (Metfor, 100 or 300 mg/kg), or Feno (50 mg/kg) + Metfor (50 mg/kg). Data are presented as means ± SEM (*n* = 6–14 rats/group). ^A^ *P* < 0.05 versus CTSH-Vehicle, ^B^ *P* < 0.05 versus DBSH-Vehicle, ^C^ *P* < 0.05 versus CTI/R-Vehicle, and ^D^ *P* < 0.05 versus DBI/R-Vehicle two-way ANOVA followed by Duncan's* post hoc* test.

**Figure 7:** Effect of the treatments on Cu/ZnSOD and MnSOD activity, evaluated in ischemic left ventricle area from control- (CT-) and diabetic- (DB-) rats subjected to sham- (SH-) or ischemia/reperfusion- (I/R-) myocardial infarction and treated subchronically (14 d) with either vehicle, fenofibrate (Feno, 100 mg/kg), metformin (Metfor, 100 or 300 mg/kg), or Feno (50 mg/kg) + Metfor (50 mg/kg). (a) Cu/ZnSOD and (b) MnSOD activity (*n* = 4–6 rats/group). ^A^ *P* < 0.05 versus CTSH-Vehicle, ^B^ *P* < 0.05 versus DBSH-Vehicle, ^C^ *P* < 0.05 versus CTI/R-Vehicle, and ^D^ *P* < 0.05 versus DBI/R-Vehicle two-way ANOVA followed by Duncan's* post hoc* test. Data are presented as means ± SEM.

**Figure 8:** Subchronic treatment with fenofibrate (F), metformin (M), and their combination increases GTPCH-I expression and BH_4_ : BH_2_ ratio in both control- (CT-) and diabetic- (DB-) rats subjected to ischemia/reperfusion (I/R). GTPCH-I expression was evaluated in ischemic left ventricle area from CT- and DB-rats subjected to sham- (SH-) or I/R-myocardial infarction and treated subchronically (14 d) with either vehicle, fenofibrate (F, 100 mg/kg), metformin (M, 100 or 300 mg/kg), or Feno (50 mg/kg) + Metfor (50 mg/kg). (a) Representative immunoblot and GTPCH-I expression (*n* = 4 rats/group) and (b) BH_4_ : BH_2_ ratio (*n* = 4–6 rats/group). ^A^ *P* < 0.05 versus CTSH-Vehicle, ^C^ *P* < 0.05 versus CTI/R-Vehicle, and ^D^ *P* < 0.05 versus DBI/R-Vehicle two-way ANOVA followed by Duncan's* post hoc* test. Data are presented as means ± SEM.

**Figure 9:** Effect of fenofibrate, metformin, and their combination on nitric oxide system. (a) The expression of endothelial nitric oxide synthase (eNOS) was analyzed by Western blot in the left ventricle of control- (CT-) and diabetic- (DB-) rats, subjected to sham (SH) or ischemia/reperfusion (I/R) injury, receiving 14 days of either vehicle, fenofibrate (F or Feno, 100 mg/kg), metformin (M or Metfor, 100 or 300 mg/kg), or Feno (50 mg/kg) + Metfor (50 mg/kg) and (b) tissue NO production and the activity of (c) eNOS and (d) iNOS. The bars represent the mean ± SEM of 4–6 different experiments. ^A^ *P* < 0.05 versus CTSH-Vehicle, ^B^ *P* < 0.05 versus DBSH-Vehicle, ^C^ *P* < 0.05 versus CTI/R-Vehicle, and ^D^ *P* < 0.05 versus DBI/R-Vehicle two-way ANOVA followed by Duncan's* post hoc* test.
